The article "The therapeutic efficacy of transcranial magnetic stimulation in managing Alzheimer’s disease: A systemic review and meta-analysis" was published in 2022. Journal: Front Aging Neurosci.

# The therapeutic efficacy of transcranial magnetic stimulation in managing Alzheimer’s disease: A systemic review and meta-analysis

**DOI:** 10.3389/fnagi.2022.980998

**Published:** 2022-09-06

**Authors:** Zhenyu Wei, Jiaqi Fu, Huazheng Liang, Mingli Liu, Xiaofei Ye, Ping Zhong

**Affiliations:** ^1^Department of Neurology, Shidong Hospital Affiliated to University of Shanghai for Science and Technology, Shanghai, China; ^2^School of Health Science and Engineering, Shanghai University of Science and Technology, Shanghai, China; ^3^Clinical Research Center for Anesthesiology and Perioperative Medicine, Shanghai Fourth People’s Hospital, School of Medicine, Tongji University, Shanghai, China; ^4^Translational Research Institute of Brain and Brain-Like Intelligence, Shanghai Fourth People’s Hospital, School of Medicine, Tongji University, Shanghai, China; ^5^Department of Statistics, Naval Medical University, Shanghai, China

**Keywords:** repetitive transcranial magnetic stimulation, Alzheimer’s disease, cognitive function, activities of daily living, therapeutic efficacy

## Abstract

**Background:**

Repetitive Transcranial Magnetic Stimulation (rTMS) is widely used to treat Alzheimer’s Disease. However, the effect of rTMS is still controversial. The purpose of the present study is to evaluate the effectiveness of rTMS on cognitive performance of AD patients.

**Methods:**

We systematically searched relevant literatures in four major databases - PubMed, EMBASE, Web of Science, and the Cochrane Central Register of Controlled Trials [Central] before 28*^th^* April 2022. Both randomized controlled trials and cross-section studies that compared the therapeutic effect of rTMS with blank control or sham stimuli were included.

**Results:**

A total of 14 studies involving 513 AD patients were finally included for meta-analysis. It was found that rTMS significantly improved global cognitive function (SMD = 0.24, 95%CI, 0.12 to 0.36, *P* = 0.0001) and daily living ability (IADL: SMD = 0.64, 95%CI, 0.21to 1.08, *P* = 0.004) in patients with AD, but did not show improvement in language, memory, executive ability, and mood. In further analyses, rTMS at 10 Hz, on a single target with 20 sessions of treatment was shown to produce a positive effect. In addition, improvement in cognitive functions lasted for at least 6 weeks (SMD = 0.67, 95%CI, 0.05 to 1.30,*P* = 0.04).

**Conclusion:**

rTMS can improve the global cognition and daily living ability of AD patients. In addition, attention should be paid to the safety of rTMS in AD patients with seizures. Given the relatively small sample size, our results should be interpreted with caution.

## Introduction

Dementia is an acquired, progressive cognitive impairment that affects the activities of daily living and is one of the leading causes of dependency, disability, and death. Currently, there are approximately 44 million patients inflicted by dementia in the world and the number of patients is estimated to triple by 2050 as the aging population increases (Lane et al., 2018). Alzheimer’s disease (AD) is the predominant cause of dementia, accounting for 50–75% of dementia patients. Its incidence nearly doubles every 5 years after the age of 65 (Albanese et al., 2014). Clinically, it manifests mainly in cognitive impairment, abnormal psychomotor behaviors and social withdrawal, which significantly increase the risk of emotional distress and negative physical and mental health consequences (Alzheimer’s Association, 2021). Currently, there are five FDA approved medications to treat AD, including acetylcholinesterase inhibitors and a glutamate receptor antagonist (memantine) (Raina et al., 2008). Given the limited effect of existing pharmacological therapies for restoring brain functions, clinicians and researchers are looking for answers in the field of non-pharmacological interventions. As a non-invasive intervention, transcranial magnetic stimulation (TMS) may improve neuroplasticity and cognitive function. It is increasingly considered as a potential therapeutic strategy for the treatment of AD.

The article "The therapeutic efficacy of transcranial magnetic stimulation in managing Alzheimer’s disease: A systemic review and meta-analysis" was published in 2022. Journal: Front Aging Neurosci.

Transcranial magnetic stimulation (TMS) is a non-invasive neuromodulation technique. Its magnetic pulses cross the thickness separating the surface of the skin to the surface of the brain. Variation in the intensity of the magnetic field induces electric fields which can stimulate specific brain regions (Liao et al., 2015). It can regulate not only the excitability of nerves and functions of the cortices (Gangitano et al., 2002), but also the activity of individual neurons (Mueller et al., 2014). Therefore, it has been widely used to treat depression, pain, fibromyalgia, post-traumatic stress disorder, non-fluent aphasia after stroke (Lefaucheur et al., 2020), and cognitive impairment (Trung et al., 2019). Though many clinical trials have investigated the efficacy and safety of repetitive TMS (rTMS) for patients with AD (Cotelli et al., 2011; Ahmed et al., 2012; Koch et al., 2018), and a number of meta-analyses have been published (Dong et al., 2018; Lin et al., 2019; Wang et al., 2020; Teselink et al., 2021), no consensus has been reached. A recent meta-analysis summarized results from randomized controlled trials published in PubMed and Web of Science, but the impact of single point stimulation, multi-point stimulation, the number of sessions of treatment, and combined treatment with cognitive training on AD was not reported. Therefore, we conducted this systematic review and meta-analysis on all RCT and cross-section studies published by 28*^th^* April 2022 aiming to draw a clear conclusion on the efficacy of rTMS in managing AD from multiple perspectives. The impact of rTMS on both global cognitive functions and different cognitive domains was also analyzed.

The article "The therapeutic efficacy of transcranial magnetic stimulation in managing Alzheimer’s disease: A systemic review and meta-analysis" was published in 2022. Journal: Front Aging Neurosci.

## Materials and methods

The present study was conducted by complying with the PRISMA guideline for systematic evaluation and meta-analysis (McInnes et al., 2018). This study was registered at PROSPERO^1^.

### Literature searching strategy

Two researchers (Wei and Fu) independently searched literatures on PubMed, EMBASE, Web of Science, and the Cochrane Central Register of Controlled Trials [Central] using the following keywords: (“Alzheimer’s Disease” or “Dementia of Alzheimer type” or “AD”) and (“transcranial magnetic stimulation” or “repetitive transcranial magnetic stimulation” or “TMS” or “rTMS”) and (“randomized controlled trial” OR “controlled clinical trial” OR “cross-section” OR randomized OR placebo OR “drug therapy” OR randomly OR trial OR groups). Among these publications, randomized controlled studies and cross-section studies published before or on 28*^th^* April, 2022 were selected. If there was any inconsistency between the two researchers, a senior investigator (Zhong) was invited to determine whether to include the articles against the inclusion and exclusion criteria and to approve the final list of articles.

### Eligibility criteria

Eligibility criteria were: all full-text randomized controlled studies and cross-section studies published in English, according to the National Institute of Neurological and Communicative Disorders and Stroke and the Alzheimer’s Disease and Related Disorders Association (NINCDS-ADRDA), the Diagnostic and Statistical Manual of Mental Disorders 5th Edition (DSM V) or 4th Edition (DSM IV), rTMS was administered to an age – and sex-neutral population diagnosed with AD. For specific cortical regions, rTMS was the only different intervention, while sham rTMS in the same cortical regions was defined as control conditions. Global cognition, as measured by objective (rather than subjective) cognitive scales, or any changes between baseline and post-intervention in any cognitive domains were considered as cognition-related neurobehavioral outcomes. If an article was present in multiple databases, the one containing more patients or more detailed information was included. If relevant results were reported at different time points, those from the most recent time point was used.

### Data extraction

Two researchers independently extracted the following information from each included study: authors, year of publication, research type, population characteristics (like age, sex ratio, years of education, the course of the disease, diagnosis criteria), type and characteristics of stimuli (including intensity, frequency, site, sessions of treatment), neurobehavioral outcomes [mean and standard deviation (SD)], and adverse events. Quality assessments of included studies were extracted from studies. For cross-design clinical studies, we extracted changes in outcomes before and after treatment in a single group. For clinical studies with multiple treatment groups, results were pooled and analyzed. When the Mean and SD were not shown in the text, corresponding authors were contacted for this information. If the author did not respond, measurements were taken from figures available in the article using WebPlot Digitizer-Copyright 2010-2021 Ankit Rohatgi. If any of these measures failed, the article was excluded.

The article "The therapeutic efficacy of transcranial magnetic stimulation in managing Alzheimer’s disease: A systemic review and meta-analysis" was published in 2022. Journal: Front Aging Neurosci.

### Quality assessment

According to the evaluation criteria of the Cochrane risk of bias tool (Sterne et al., 2019), two researchers (Wei and Fu) assessed the quality of methods adopted by included studies. Any disagreement was resolved through discussion or by inviting a senior researcher. Quality assessment for each study included the following seven aspects: (1) random sequence generation; (2) allocation concealment; (3) blinding of participants and implementers; (4) blinding of outcome assessment; (5) integrity of results; (6) selective reporting; (7) other biases. The risk of bias in each aspect was categorized into three risk levels: low, high, or unclear.

### Data analysis

The CochraneRev-Man 5.4 software was used for statistical analysis of the data, calculating and reporting the standardized mean difference (SMD) and 95% confidence interval for each major outcome. SMD describes how much an intervention affects outcome, and an effect of ≥ 0.8 is considered significant and potentially clinically relevant. Reports on global cognitive functions (MMSE, MoCA, ADAS-Cog, ACE-III), language (sentence comprehension test), memory (RAVLT), the ability to execute (TMT-A), daily life ability (IADL) and emotion (GDS) were included in the meta-analysis. I^2^ was used to evaluate the heterogeneity of the included studies: when *I*^2^ < 50%, it was considered to have low heterogeneity, and the fixed-effect model was used. When I^2^ value ≥ 50%, it was considered to have high heterogeneity, and the random-effects model was used to summarize the effect size. If data from at least ten studies were available, a meta-regression analysis was performed to assess the relationship between age, scale choice, frequency of stimulation, site of stimulation, and number of sessions of treatment and TMS treatment outcomes. STATA17.0 software was used to construct funnel plots for qualitative evaluation of publication bias, Begg and Egger tests were used for quantitative evaluation. The data we used were changes in scores assessed using cognition assessment scales relative to baseline scores after completion of treatment. When score changes were not directly provided in the study, use the following formula to convert the data provided in the article:

Mean change = mean final–mean baseline


$$SDchange=\sqrt{\begin{array}{c} \mathrm{SD}{\mathrm{baseline}}^{2}+\mathrm{SD}{\mathrm{final}}^{2}-(2\times \text{coefficent}\times \mathrm{SD}\mathrm{baseline}\times \mathrm{SD}\mathrm{final}) \end{array}}$$

In all analysis, *p* < 0.05 was considered statistically significant.

The article "The therapeutic efficacy of transcranial magnetic stimulation in managing Alzheimer’s disease: A systemic review and meta-analysis" was published in 2022. Journal: Front Aging Neurosci.

## Results

### Literature screening

A total of 1,059 articles were found in 4 major databases using a variety of searching strategies. A total of 263 publications were excluded due to duplicates or incomplete basic information. Another 754 publications were excluded because they were irrelevant to the condition we were interested in, basic scientific research, or non-randomized controlled studies. When the full text was inspected, 2 were excluded because of the single arm nature, 5 because of inconsistent control measures were taken, 2 because of inconsistent outcome indices, 4 because of meeting summaries or reviews, 8 because of incomplete data, another 7 because they were study protocols. Finally, 14 articles were selected for meta-analysis (Figure 1).

**FIGURE 1:** Diagram of literature searching and selection for meta-analysis.

### Information of included studies

A total of 513 AD patients with varying degrees of severity were included in this meta-analysis. Their age ranged from 60 to 80 years and 53.5% of them were female. Demographic information of the participants was summarized in Table 1, types and characteristics of the stimuli in Table 2. Sham-rTMS was similar to the real rTMS in sound and feeling upon contacting with the head, but did not produce actual therapeutic effects. Generally, the coil was tilted away from the head to achieve the purpose of false stimulation. For example, in the study of Jia et al. (2021), the same coil was tilted 45° from the scalp so that one side of the coil was in contact with the scalp and the distance between the center of the coil and the target site was greater than 5 cm. Patients would also feel the noise and sensation caused by the same stimulation. In the study of Wu et al. (2015), the coil was flipped 180°, where the coil was perpendicular to the scalp in the study of Zhang et al. (2019). In other studies, special fake coil was used, or the coil was attached to the scalp, but no therapeutic stimuli were applied.

The article "The therapeutic efficacy of transcranial magnetic stimulation in managing Alzheimer’s disease: A systemic review and meta-analysis" was published in 2022. Journal: Front Aging Neurosci.

**TABLE 1:** Demographic characteristics of included trials.

No.	Study (time)	Design	Participants (N)	Sex (M/F)	Mean age (years)	Mean education (years)	Mean disease duration (year)	Diagnostic criteria
1	Ahmed et al. (2012)	Parallel	rTMS-20HZ(15)	5/10	65.9	NA	3.9	NINCDS-ADRDA
			rTMS-1HZ(15)	6/9	68.6	NA	4.1	
			Sham(15)	5/10	68.3	NA	4.4	
2	Li et al. (2021)	Parallel	rTMS (37)	20/17	66	5.7	3.7	DSM-V
			Sham(38)	24/14	64.6	6.6	3.97	
3	Cotelli et al. (2011)	Parallel	rTMS(5)	NA	71.2	6.4	NA	NINCDS-ADRDA
			Sham(5)	NA	74.4	4.8	NA	
4	Jia et al. (2021)	Parallel	rTMS(35)	10/25	71.4	7.7	NA	DSM-V
			Sham(34)	11/23	73.4	7.5	NA	
5	Leocani et al. (2020)	Parallel	rTMS(16)	9/7	69.6	9.2	4.2	NINCDS-ADRDA
			Sham(12)	6/6	72.6	7.8	4.2	
6	Padala et al. (2020)	Parallel	rTMS(9)	8/1	74.3	NA	NA	NA
			Sham(11)	10/1	79.6	NA	NA	
7	Rabey et al. (2013)	Parallel	rTMS-COG(7)	5/2	72.6	NA	NA	DSM-V
			Sham(8)	5/3	75.4	NA	NA	
8	Wu et al. (2015)	Parallel	rTMS(26)	10/16	71.4	11.4	5.1	NINCDS-ADRDA
			Sham(26)	11/15	71.9	11.5	5.1	
9	Zhang et al. (2019)	Parallel	rTMS-COG(15)	3/12	69	12.4	3.53	NINCDS-ADRDA
			Sham(13)	3/10	68.5	11.9	3.62	
10	Zhao et al. (2017)	Parallel	rTMS(17)	7/10	69.3	4.8	NA	DSM-IV
			Sham(13)	6/7	71.4	4.9	NA	
11	Bagattini et al. (2020)	Parallel	rTMS-COG(27)	17/10	73.56	8.85	1.94	NA
			Sham(23)	12/11	73.35	7.91	1.67	
12	Koch et al. (2018)	Cross-section	rTMS/sham(14)	7/7	70	7.2	NA	NA
							NA	
13	Turriziani et al. (2019)	Parallel	rTMS(7)	5/9	71.28	14.28	NA	NA
			Sham(7)		71.71	13	NA	
14	Vecchio et al. (2022)	Parallel	Real rTMS-COG(30)	14/16	71.07	13.87	NA	NA
			Sham rTMS-COG(17)	10/7	72.24	11.47	NA	
			Sham(16)	5/11	75.2	11.81	NA	

No, number; M, male; F, female; COG, cognitive training; NA, not reported.

**TABLE 2:** Description of repetitive transcranial magnetic stimulation (rTMS) intervention in the included studies.

No.	Study (time)	Groups	Frequency	Stimulation protocol	Stimulation sites	Number of sessions	Length of follow-up
1	Ahmed et al. (2012)	rTMS-20HZ	20 Hz	90% of MT, 2000 pulses	L/R-DLPFC	5	4 and 12 weeks.
		rTMS-1HZ	1 Hz	100% of MT,2000 pulses			
		sham	\	the coil angled away from the head			
2	Li et al. (2021)	rTMS	20 Hz	100% of MT, 2000 pulses	L-DLPFC	30	12 weeks
		sham	\	used a pseudo-stimulus coil			
3	Cotelli et al. (2011)	rTMS	20 Hz,	100% of MT, 2000 pulses	L-DLPFC	10	8 weeks
		sham	\	used a sham coil			
4	Jia et al. (2021)	rTMS	10 Hz	100–110% of MT, 800 pulses	left lateral parietal cortex site	10	NA
		sham	\	the coil was rotated 45?away from the brain			
5	Leocani et al. (2020)	rTMS	10 Hz	120% of MT, 840 pulses	bilateral frontalparietal-temporal regions	16	NA
		sham	\	used a sham coil			
6	Padala et al. (2020)	rTMS	10 Hz	120% of MT, 3000 pulses	L-DLPFC	20	8 and 12 weeks
		sham	\	NA			
7	Rabey et al. (2013)	rTMS-COG	10 Hz	90–110 % of MT, 1300 pulses	Broca, Wernicke, L/R-DLPFC, L/R pSAC	54	NA
		sham	\	using a sham coil			
8	Wu et al. (2015)	rTMS	20 Hz	80% of MT, 1200 pulses	L-DLPFC	20	NA
		sham	\	the coils were turned 180°			
9	Zhang et al. (2019)	rTMS-COG	10 Hz	100% of RMT, 1000 pulses	L-DLPFC	20	4 weeks
		sham	\	the coils were turned 90°			
10	Zhao et al. (2017)	rTMS	20 Hz	NA	parietal P3/P4 and posterior temporal T5/T6	30	6 weeks
		sham	\	used a sham coil			
11	Bagattini et al. (2020)	rTMS-COG	20Hz	100% of MT, 2000 pulses	L-DLPFC	20	12 weeks
		sham	\	a 3-cm thick block of wood was placed between the coil and the scalp			
12	Koch et al. (2018)	rTMS	20Hz	100% of RMT, 1600 pulses	Precuneus	10	NA
		sham	\	used a sham coil			
13	Turriziani et al. (2019)	rTMS	1Hz	90% of MT, 600 pulses	R-DLPFC	10	4 weeks
		sham	\	\			
14	Vecchio et al. (2022)	Real rTMS -COG	10Hz	90–110% of MT, 1200–1400 pulses	Broca, Wernicke, L/R-DLPFC, L/R pSAC	30	40 weeks
		Sham rTMS -COG	\	using a sham coil			
		Sham	\	using a sham coil			

L, left; R, right; DLPFC, dorsolateral prefrontal cortex; pSAC, parietal somatosensory association cortex; MT, motor threshold.

The article "The therapeutic efficacy of transcranial magnetic stimulation in managing Alzheimer’s disease: A systemic review and meta-analysis" was published in 2022. Journal: Front Aging Neurosci.

High frequency rTMS (HFrTMS) was dominantly used by included studies with 7 studies adopting high frequency up to 20 Hz (Cotelli et al., 2011; Ahmed et al., 2012; Wu et al., 2015; Zhao et al., 2017; Koch et al., 2018; Bagattini et al., 2020; Li et al., 2021). Studies by Ahmed et al compared the effects of high (20Hz) and low frequencies (1Hz) (Ahmed et al., 2012). A study by Turriziani et al. (2019) used 1 Hz, and the other 6 studies used 10 Hz (Rabey et al., 2013; Leocani et al., 2020; Padala et al., 2020; Jia et al., 2021; Vecchio et al., 2022). The dorsolateral prefrontal cortex (DLPFC) was selected as the stimulation site in the majority of studies (10/14) (Cotelli et al., 2011; Ahmed et al., 2012; Rabey et al., 2013; Wu et al., 2015; Turriziani et al., 2019; Zhang et al., 2019; Bagattini et al., 2020; Padala et al., 2020; Li et al., 2021; Vecchio et al., 2022). Rabey et al. (2013) and Vecchio et al. (2022) stimulated Broca, Wernicke, L/R-DLPFC, and L/R pSAC. Zhao et al. (2017) stimulated four parietal P3/P4 and posterior temporal T5/T6. Regarding the type of coil used for stimulation, the H-type coil was used in the study of Leocani et al. (2020), whereas the rest of the studies used the “8” shaped coil. Among the 14 studies, the majority of them adopted 10 to 30 sessions, with a maximum of 54 and a minimum of 5 sessions. A number of studies reported cognitive performance at follow-up ranging from 1 to 10 months. Four studies reported adverse reactions during the treatment (Zhang et al., 2019; Leocani et al., 2020; Padala et al., 2020; Jia et al., 2021).

The article "The therapeutic efficacy of transcranial magnetic stimulation in managing Alzheimer’s disease: A systemic review and meta-analysis" was published in 2022. Journal: Front Aging Neurosci.

### Quality of included studies

The quality of included studies was independently assessed using the Revman software by two researchers. As shown in Table 2, only the study by Koch et al. (2018) used the cross design, and the rest were randomized controlled studies. These indicate that the overall quality of the included studies was good (Figure 2).

**FIGURE 2:** Analysis of risk of bias.

### The effect of repetitive transcranial magnetic stimulation on global cognitive functions

Thirteen studies assessed the impact of rTMS on global cognitive functions, namely, the Mini-Mental State Examination (MMSE), Montreal Cognitive Assessment (MoCA), Addenbrooke’s Cognitive Examination III (ACE-III) and the Alzheimer’s Disease Assessment Scale-Cognitive Subscale (ADAS-Cog). Among these studies, 3 used the MMSE and ADAS-cog scales to assess patients’ global cognitive status (Zhao et al., 2017; Zhang et al., 2019; Li et al., 2021), 6 studies counted MMSE results (Cotelli et al., 2011; Ahmed et al., 2012; Koch et al., 2018; Bagattini et al., 2020; Padala et al., 2020; Jia et al., 2021), and 4 studies counted ADAS-cog results (Rabey et al., 2013; Wu et al., 2015; Leocani et al., 2020; Vecchio et al., 2022). The above findings showed that rTMS significantly improved global cognitive functions (measured by MMSE or ADAS-Cog) in AD patients (SMD = 0.34,95% CI, 0.16 to 0.52, *p* = 0.0002, *I*^2^ = 0%, Figure 3). When subgroup analysis was conducted to discuss MMSE and ADAS-cog, respectively, rTMS still had a significant effect on the global cognitive functions of AD patients (MMSE: SMD = 0.59, 95%CI, 0.36 to 0.81, *I*^2^ = 87%; ADAS-cog: SMD = –0.34, 95%CI, –0.59 to –0.10, *I*^2^ = 42%) (Figure 3). It should be noted that the MMSE score is a positive indicator, and the higher the score, the better the cognitive status of patients. While ADAS-cog is a negative indicator, the lower the score, the better the cognitive status of patients. In our forest map, the abscissa is defined according to the MMSE score, that is, the left is the sham stimulation group, and the right is the rTMS treatment group. However, for the subgroup analysis of ADAS-cog, we accurately calculated the results of each study, so the SMD values of subgroups that fell on the left indicated that the rTMS treatment was effective. In particular, Zhao et al. (2017) additionally used the MoCA scale to show that rTMS had a significant treatment effect [rTMS change (Mean ± SD): 2.3 ± 6.36; sham change (Mean ± SD): 1.2 ± 7.02]. Zhang et al. (2019) also observed more significant results using the ACE-III scale [rTMS change (Mean ± SE): 11.77 ± 1.32; Sham change (Mean ± SE): 2.18 ± 1.43].

The article "The therapeutic efficacy of transcranial magnetic stimulation in managing Alzheimer’s disease: A systemic review and meta-analysis" was published in 2022. Journal: Front Aging Neurosci.

**FIGURE 3:** The effect of repetitive transcranial magnetic stimulation (rTMS) on global cognitive functions.

Inconsistencies exist in the rTMS intervention parameters among the included studies, and we conducted subgroup analyses on stimulation frequency, stimulation sites, and the number of sessions of treatment. As shown in Figure 4, compared with rTMS at 20 Hz, stimulation frequency at 10 Hz had a more significant effect (SMD = 0.29, 95%CI, 0.01 to 0.57, *P* = 0.04). When analyzing the influence of stimulating loci, it was found that single stimulation of L-DLPFC (SMD = 0.84, 95%CI, 0.08 to 1.59, *P* = 0.03) was more effective than multi-point stimulation (SMD = 0.30, 95%CI, 0.00 to 0.61, *P* = 0.05) (Figure 5). In addition, the therapeutic effect was most significant when the number of treatment sessions was 20 (SMD = 0.61, 95%CI, 0.28 to 0.95, *P* = 0.0003), followed by treatment sessions over 20 (SMD = 0.39, 95%CI, 0.07 to 0.70, *P* = 0.02). No statistical difference was observed when the number of treatment sessions was less than 20 (SMD = 0.16, 95%CI, –0.12 to 0.45, *P* = 0.26) (Figure 6). Some of the studies in the meta-analysis also provided participants with supplemental cognitive training when assessing the impact of rTMS on global cognition, but the content of cognitive training varied between studies (Rabey et al., 2013; Zhang et al., 2019; Bagattini et al., 2020; Vecchio et al., 2022).

**FIGURE 4:** Impact of repetitive transcranial magnetic stimulation (rTMS) stimulation frequency on global cognitive functions.

**FIGURE 5:** Impact of repetitive transcranial magnetic stimulation (rTMS) stimulation site of rTMS on global cognitive functions.

**FIGURE 6:** Influence of sessions of repetitive transcranial magnetic stimulation (rTMS) treatment on global cognitive functions.

Our results showed that rTMS combined with cognitive training had no statistically significant effect on global cognitive functions (SMD = 0.48, 95%CI, –0.08 to 1.05, *P* = 0.09), but rTMS without combined cognitive training seemed to be superior to the former in improving global cognitive functions. The statistical significance of the results remains to be explored (SMD = 0.54, 95%CI, 0.01 to 1.06, *P* = 0.05) (Figure 7). Among the included studies, 6 reported post-treatment effects (Ahmed et al., 2012; Zhao et al., 2017; Zhang et al., 2019; Bagattini et al., 2020; Li et al., 2021; Vecchio et al., 2022). Results showed that rTMS had a better effect when the follow-up time was > 6 weeks (SMD = 0.67, 95%CI, 0.05 to 1.30, *P* = 0.04) than ≤6 weeks (SMD = 0.53, 95%CI, 0.00 to 1.05, *P* = 0.05) (Figure 8).

The article "The therapeutic efficacy of transcranial magnetic stimulation in managing Alzheimer’s disease: A systemic review and meta-analysis" was published in 2022. Journal: Front Aging Neurosci.

**FIGURE 7:** Influence of repetitive transcranial magnetic stimulation (rTMS) combined cognitive training on global cognitive functions.

**FIGURE 8:** Post-treatment effects of repetitive transcranial magnetic stimulation (rTMS) on global cognitive functions.

### Influence of repetitive transcranial magnetic stimulation on daily living

Among the studies we included, 3 (Cotelli et al., 2011; Ahmed et al., 2012; Padala et al., 2020) analyzed daily living using the IADL scale. Their results showed that rTMS could significantly improve the daily living ability of AD patients (SMD = 0.64, 95%CI: 0.21–1.08, *P* = 0.007) (Figure 9).

**FIGURE 9:** Forest plot showing the effect of repetitive transcranial magnetic stimulation (rTMS) on IADL of AD patients with 95% CI.

### Impact of repetitive transcranial magnetic stimulation on language

In the study of Cotelli et al. (2011), the sentence comprehension test was used to evaluate the listening comprehension of AD patients, and the results showed that rTMS had a significant therapeutic effect on language. In contrast, in the study of Jia et al. (2021), the language results of the MMSE scale did not show significant improvement. In the study by Zhang et al. (2019), although the therapeutic effect of rTMS on language was observed by the ACE-III scale, the result was not statistically significant (*P* = 0.08). In addition, Zhao et al. (2017) showed significant improvement in speech function in patients treated with rTMS, and the results were statistically significant (*P* = 0.003). However, it was not clearly explained in this study how the language function score was obtained. According to the research content of Zhao et al. (2017), we inferred that the conclusion was obtained by comprehensive calculation of the results of ADAS-cog, MMSE, MoCA and WHO-UCLA AVLT scale.

### Impact of repetitive transcranial magnetic stimulation on memory

Koch et al. (2018) and Bagattini et al. (2020) used RAVLT-IR and RAVLT-DR tests to evaluate the memory function of patients. Since both tests belong to the RAVLT subscale and they are strongly correlated, so the results of these two tests were combined for analysis. However, the rTMS group did not show superiority to the sham stimulation group (SMD = 0.22, 95%CI, –0.09 to 0.54, *P* = 0.17) (Figure 10). In addition, Turriziani et al. (2019) found that AD patients did not show any difference in the Rey’s 15 words immediate recall and Rey’s 15 words 15-min delayed recall. However, a study by Zhang et al. (2019) showed that rTMS significantly improved the memory function in patients who received cognitive training [real TMS-CT change (Mean ± SE): 3.87 ± 0.82; Sham TMS-CT change (Mean ± SE): 0.29 ± 1.07]. A note is that this conclusion was drawn from ACE-III results.

The article "The therapeutic efficacy of transcranial magnetic stimulation in managing Alzheimer’s disease: A systemic review and meta-analysis" was published in 2022. Journal: Front Aging Neurosci.

**FIGURE 10:** Forest plot showing the effect of repetitive transcranial magnetic stimulation (rTMS) on RAVLT of AD patients with 95% CI.

### Impact of repetitive transcranial magnetic stimulation on executive ability

In studies by Bagattini et al. (2020) and Padala et al. (2020), rTMS showed no positive effect when the “Visuospatial Ability” and “Writing Movement Speed” were evaluated using the TMT A test (SMD = 0.02, 95%CI, –0.45 to 0.50, *P* = 0.93) (Figure 11). However, a positive trend was observed in a study by Zhang et al. (2019) on attention and visuospatial function assessed using the ACE-III scale.

**FIGURE 11:** Forest plot showing the effect of repetitive transcranial magnetic stimulation (rTMS) on TMT-A of AD patients with 95% CI.

### Influence of repetitive transcranial magnetic stimulation on emotion

Studies by Ahmed et al. (2012) and Bagattini et al. (2020) assessed psychological and emotional changes of AD patients using the GDS scale. It can be seen from the forest plot, there was no statistical difference in psychological and emotional improvement between the TMS treatment group and the sham stimulation group (SMD: –0.16, 95%CI: –0.54∼0.22, *P* = 0.41) (Figure 12). In another study by Padala et al. (2020), Clinical Global Impression-improvement (CGI-I) and Clinical Global Impression-Severity (CGI-S) were used to assess the overall mental state of AD patients. It was found that rTMS treatment significantly improved mental state as shown by CGI-S [1.4 (0.5 to 2.3), *P* = 0.005]. In the rTMS group, CGI-S was significantly better compared to that of the baseline (*P* < 0.001), whereas no significant difference was found between the baseline and after sham stimulation (*P* = 0.238) in the sham group. In contrast, when CGI-I was used to assess psychological and emotional changes [–2.56 (–3.5 to –1.6), *P* < 0.001], both rTMS and sham stimulation significantly improved CGI-I compared to the baseline.

**FIGURE 12:** Forest plot showing the effect of repetitive transcranial magnetic stimulation (rTMS) on GDS of AD patients with 95% CI.

### Publication bias and sensitivity analysis

We first used funnel plots to qualitatively assess publication bias, and our results showed that funnel plots were visually symmetric (Figure 13). Then we conducted quantitative evaluation through Begg and Egger tests, and results showed that publication bias was present [Begg (*P* = 0.0748) and Egger (*P* = 0.0040)]. Therefore, pruning and filling tests were used for verification. After pruning and filling, our results did not change, suggesting that they were still robust (Figure 13). In addition, it should be pointed out that the methods of random sequence generation and concealment in the study by Cotelli et al. (2011) were not reported, suggesting a highly potential bias risk (Figure 2). After excluding this study, the influence of rTMS on AD patients (SMD = 0.57; 95% CI = 0.39, 0.76; *P* < 0.00001, *I*^2^ = 83%) was still significantly higher than those in the sham stimulation group. We then conducted a sensitivity analysis using the leave one method, iteratively deleting each study and recalculating the summary SMD. The data showed that the heterogeneity of the results changed significantly when the study of Li et al. (2021) was excluded alone. But the results were still statistically significant (SMD = 0.36, 95%CI = 0.17–0.55; *P* = 0.0002, *I*^2^ = 54%). Meta-regression analysis was used to explore the source of heterogeneity, and the results showed that sample size, age and TMS treatment effect were not significant at the level of 5%, that is, sample size and age were not considered as the source of heterogeneity (sample size: *P* = 0.177; age: *P* = 0.952). Scale selection and TMS treatment effect were significant at the level of 1%, stimulation frequency was significant at the level of 5%. We have conducted subgroup analysis on rTMS stimulation frequency, number of stimulation sites, and number of sessions using different cognitive scales.

The article "The therapeutic efficacy of transcranial magnetic stimulation in managing Alzheimer’s disease: A systemic review and meta-analysis" was published in 2022. Journal: Front Aging Neurosci.

**FIGURE 13:** Funnel plot for publication bias and result of clipping test.

### Adverse reactions

Adverse reactions were reported in 4 of 14 studies (Zhang et al., 2019; Leocani et al., 2020; Padala et al., 2020; Jia et al., 2021). The main adverse reactions included local scalp discomfort or headache. In a study by Jia et al. (2021), two patients (one in the rTMS group and the other in the sham group) reported transient fatigue. It has to be mentioned that no case of seizure was recorded.

## Discussion

The present study included 14 studies, involving a total of 513 AD patients with varying degrees of disease severity, comparing the improvement of cognitive performance after rTMS treatment or sham stimulation. We found that rTMS significantly improved global cognitive functions compared to sham stimulation. When each cognitive domain was taken into account for further analysis, we found that rTMS was effective in improving the performance in daily living ability. Our results are consistent with most previous reports that rTMS has a positive impact on cognition and daily living of AD patients.

The article "The therapeutic efficacy of transcranial magnetic stimulation in managing Alzheimer’s disease: A systemic review and meta-analysis" was published in 2022. Journal: Front Aging Neurosci.

Previous studies have proven that the cortical plasticity of AD patients is impaired (Di Lorenzo et al., 2020), leading to decline of cognitive functions and self-care ability (Di Lorenzo et al., 2019), rTMS can improve the plasticity and excitability of the cerebral cortex (Pennisi et al., 2011), and consequently improve the cognitive performance of AD patients. Though our study is unable to test neural plasticity, the improved performance in global cognitive functions and some of the domains suggests that rTMS may improve neural plasticity.

Cognitive impairment includes alterations in executive, visuospatial, speech, memory and other aspects. Our meta-analysis showed that rTMS can improve global cognitive functions in patients with AD, which is consistent with findings of a previous meta-analysis study (Lin et al., 2019). Thirteen of our included studies assessed global cognitive functions in patients with AD using scales, such as MMSE, MoCA, ACE-III and ADAS-cog with consistent and positive results (Cotelli et al., 2011; Ahmed et al., 2012; Rabey et al., 2013; Wu et al., 2015; Koch et al., 2018; Zhang et al., 2019; Bagattini et al., 2020; Leocani et al., 2020; Padala et al., 2020; Jia et al., 2021; Li et al., 2021; Vecchio et al., 2022). Although individual studies in our included studies showed positive results in the areas of language, memory, executive function, and emotional cognition, the combined results were not statistically significant. Language is a tool to communicate with symbols. The three elements of language include pronunciation, semantics, and grammar. Verbal communication plays a central role in human social interaction. Language impairment is one of the common functional impairments in cognitive impairment and appears in the early stage of AD. Language task performance is an important diagnostic criterion for AD and mild cognitive impairment.

It is mainly manifested in language fluency, naming, semantic knowledge, and discourse processing (Taler and Phillips, 2008). The language assessment Scale is a commonly used method for the assessment of language disorders, including aphasia screening test, Boston Naming test, Word Fluency test, double-listening test, expression vocabulary test, Peabody Graph word test, adult reading test, marking test, and language test of Wechsler Intelligence Test. In previous studies, there were few articles related to rTMS research on the language cognitive domain of AD patients, and the assessment methods used in the study were not uniform, which made it difficult to conduct further statistical analysis. Therefore, we described the relevant articles one by one. Cotelli et al. (2011) evaluated the patients’ listening comprehension ability through the Sentence Comprehension test and obtained positive results. However, in the study of Zhang et al. (2019) and Jia et al. (2021), the results of language function measured by MMSE and ACE-III, respectively, were not statistically significant. In the study of memory cognitive domain, Koch et al. (2018) and Bagattini et al. (2020) used RAVLT as an evaluation tool to conduct the study, and the results showed that there was no significant statistical difference between the TMS treatment group and the sham stimulation control group. In terms of executive ability, Bagattini et al. (2020) and Padala et al. (2020) did not show positive effects of rTMS when TMT A test was used to evaluate “visuospatial ability” and “writing motor speed.” However, Zhang et al. (2019) observed positive results in “attention” and “visuospatial ability” using the ACE-III scale.

The article "The therapeutic efficacy of transcranial magnetic stimulation in managing Alzheimer’s disease: A systemic review and meta-analysis" was published in 2022. Journal: Front Aging Neurosci.

In the population aged 65 and over, 35% suffer from disabilities, such as decreased activities of daily living (ADL) and instrumental ADL (IADL), which may make it difficult for elderly people to live independently (Kiyoshige et al., 2019). IADL represents the ability to use public transportation, buy daily necessities, prepare meals, pay bills, manage bank accounts, etc (Koyano et al., 1991), which means that IADL is a key factor for independent living, social interaction, and health of the elderly, and relates to the degree of autonomy and independence of an individual to engage in activities in the community and home. In terms of daily living ability, positive results were found in IADL indicators in studies of Cotelli et al. (2011); Ahmed et al. (2012), and Padala et al. (2020).

Previous studies have found that rTMS treatment has definite effects on depression and other psychiatric disorders (Health Quality Ontario, 2016; De Risio et al., 2020). In a study on the effect of rTMS on patients with treatment-refractory depression, positive response of patients was related to the increased volume of the left amygdala and the unchanged volume of the hippocampus, whereas the neutral response was associated with the decreased volume of the left hippocampus (Furtado et al., 2013). Another study reported that an increase in the volume of that the hippocampus on the side of that the brain targeted by HFrTMS was associated with improvement in depression (Hayasaka et al., 2017). However, when we analyzed combined results of GDS indicators of Ahmed et al. (2012) and Bagattini et al. (2020), we did not obtain positive results that rTMS treatment could improve the mood of AD patients. Given the small number of included studies and the different scales used in different studies, it is necessary to conduct high-quality larger-sample RCT studies in the future to confirm our findings.

The article "The therapeutic efficacy of transcranial magnetic stimulation in managing Alzheimer’s disease: A systemic review and meta-analysis" was published in 2022. Journal: Front Aging Neurosci.

Our meta-analysis also examined the effect of different rTMS parameters on cognitive performance and found that 10 Hz rTMS, 20 sessions or more, and L-DLPFC were effective in improving cognitive functions. Our results support findings of previous studies regarding the impact of different stimulation frequencies, locations, and sessions of rTMS on cognitive performance (Nguyen et al., 2017). Due to the difference in stimulation parameters, rTMS can enhance or inhibit the excitability of specific areas of the cerebral cortex (Nguyen et al., 2017; Jiang et al., 2022). In our study, 10 Hz rTMS showed a better therapeutic effect on cognitive functions, implying that HFrTMS may increase the excitability of neural cells with a ceiling effect. Considering the opposite result from a meta-analysis study by Wang et al. (2020), which claimed that 20 Hz rTMS seemed to be more effective than 10 Hz or 1 Hz rTMS, future high-quality larger-sample RCT studies are needed to draw an exclusive conclusion.

Selection of stimulating sites is a prerequisite for rTMS. The most common choices for single-site stimulation were the L-DLPFC and the Precuneus (Nardone et al., 2014; Koch et al., 2018). As mentioned above, frequency of 10 Hz had the best efficacy compared to 20 Hz, suggesting a relationship between the frequency of rTMS and the site of stimulation. The most common choice for multisite stimulation is the left and right DLPFC. Whether bilateral DLPFC stimulation is superior to unilateral DLPFC stimulation remains controversial. In a meta-analysis published by Liao et al. (2015) involving 94 patients with mild to moderate AD, it was found that stimulation of the right or bilateral DLPFC was more superior to stimulation of the L-DLPFC alone. In contrast, meta-analysis by Drumond Marra et al. (2015) and Wu et al. (2015) found that stimulation of the L-DLPFC by HFrTMS was more effective in improving cognitive performance than multi-point stimulation. Cotelli et al. (2011) found that stimulation of the L-DLPFC significantly increased the percentage of correct response in auditory sentence comprehension, but there was no significant difference in other language abilities or memory. This study only included 10 patients. To draw a clear conclusion on the efficacy of different parameters of rTMS in improving cognitive performance in diverse domains, the long-term results of studies adopting multisite stimulation are needed.

In addition, we also conducted a subgroup analysis on the effect of cognitive training added to rTMS, and we found that cognitive training did not show additive effects when applied with rTMS. But the cognitive training varied from study to study. For example, Zhang et al. (2019) adopted cognitive training in areas of memory tasks, attention tasks, mathematical calculations, agility drills and logic thinking tasks. Rabey et al. (2013) and Vecchio et al. (2022) applied cognitive training to test the impact of Broca region, Wernicke region, R-DLPFC, L-DLPFC, R-PSAC, and the L-PSAC on cognitive performance. Cognitive training in the study by Bagattini et al. (2020) focused on episodic memory and specifically on face-name associative memory. Although the above studies separately described the positive results of rTMS combined with cognitive training, our results did not show statistical significance in our subgroup analysis (SMD = 0.48, 95%CI: –0.08 to 1.05, *P* = 0.09). Therefore, future studies should balance the number of AD patients receiving the combined cognitive training and those who do not receive this combined therapy, in order to better investigate whether cognitive training leads to synergistic effects.

The article "The therapeutic efficacy of transcranial magnetic stimulation in managing Alzheimer’s disease: A systemic review and meta-analysis" was published in 2022. Journal: Front Aging Neurosci.

In the study of Zhang et al. (2019), MMSE and ACE-III indicators were used to observe the effect of rTMS 4 weeks after rTMS treatment, and the results showed that patients treated with rTMS still maintained significant improvement in cognitive functions. Zhao et al. (2017) reported the effect of rTMS 6 weeks after rTMS treatment, three cognitive domains of memory, language, and executive ability were individually analyzed based on ADAS-cog, MMSE, MoCA, and WHO-UCLA AVLT indicators. The results showed that memory function improved the most, followed by language function. Ahmed et al. (2012) reported the effect of rTMS on AD patients 1 and 3 months after rTMS treatment, respectively. MMSE results showed that mild or moderate AD patients who received HFrTMS stimulation benefited the most. Positive results of long-term therapeutic effects of rTMS were reported in studies by Bagattini et al. (2020), Li et al. (2021), and Vecchio et al. (2022). Their follow-up duration was 2, 3, and 4 months, respectively. In our subgroup analysis, patients who received rTMS still maintained good cognitive function improvement within 6 weeks after the end of treatment, but the improvement effect was more apparent after over 6 weeks, evidenced by results of Ahmed et al. (2012).

Our study was conducted on the basis of the study by Lin et al. (2019), apart from global cognitive functions, different cognitive domains such as language, memory, executive ability, daily living ability and emotion, as well as rTMS parameters were analyzed, and compared at different follow-up time points. The forest maps of MMSE and ADAS-cog were drawn for analysis. In terms of publication bias and sensitivity analysis, we conducted more comprehensive validation and discussion, and the results were robust. Meta-regression analysis was used to explore the source of heterogeneity, and the results suggested that there was no correlation between sample size, age, and the therapeutic effect of rTMS.

The article "The therapeutic efficacy of transcranial magnetic stimulation in managing Alzheimer’s disease: A systemic review and meta-analysis" was published in 2022. Journal: Front Aging Neurosci.

Some limitations should be considered when interpreting our results. The use of different scales to measure global cognitive functions in different studies may lead to high heterogeneity. Meta-regression analysis suggested that scale selection was significantly associated with TMS treatment effect at the level of 1% and stimulus frequency at the level of 5%. Among the included studies, only 6 explored the therapeutic effect 1 to 3 months after completing the treatment, longer follow-up period is needed to examine the long-term therapeutic effect of rTMS on AD in the future.

## Conclusion

Repetitive transcranial magnetic stimulation (rTMS) can improve global cognitive functions and daily living ability of AD patients. Subgroup analysis showed that rTMS significantly improved cognition with 20 sessions or more at a specific single point at high frequency. In addition, we should pay more attention to the safety of rTMS in AD patients with seizures. Given the relatively small sample size, our results should be interpreted with caution. Additional studies with larger sample sizes and longer follow-up period are needed to better assess the efficacy of rTMS in managing AD patients and the optimal type of stimulation required to maximize beneficial outcomes.

## Author contributions

PZ: conceptualization, reviewing and editing, and supervision. ZW and JF: methodology, software, visualization, investigation, and original draft preparation. HL: visualization and writing—reviewing and editing. ML: literature search, methodology, software, and visualization. XY: data curation, visualization, and investigation. All authors contributed to the article and approved the submitted version.

## Footnotes

1
https://www.crd.york.ac.uk/prospero/display_record.php?ID=CRD42018089990

## References

[B1] AhmedM. A.DarwishE. S.KhedrE. M.El SerogyY. M.AliA. M. (2012). Effects of low versus high frequencies of repetitive transcranial magnetic stimulation on cognitive function and cortical excitability in Alzheimer’s dementia. *J. Neurol.* 259 83–92. 10.1007/s00415-011-6128-4 21671144

[B2] AlbaneseE.GuerchetM.PrinceM.PrinaM. (2014). *World Alzheimer Report 2014: Dementia and Risk Reduction. An Analysis of Protective and Modifiable Factors.* London: Alzheimer’s Disease International.

The article "The therapeutic efficacy of transcranial magnetic stimulation in managing Alzheimer’s disease: A systemic review and meta-analysis" was published in 2022. Journal: Front Aging Neurosci.

[B3] Alzheimer’s Association (2021). Alzheimer’s disease facts and figures. *Alzheimers Dement* 17 327–406. 10.1002/alz.12328 33756057

[B4] BagattiniC.ZanniM.BaroccoF.CaffarraP.BrignaniD.MiniussiC. (2020). Enhancing cognitive training effects in Alzheimer’s disease: rTMS as an add-on treatment. *Brain Stimul.* 13 1655–1664. 10.1016/j.brs.2020.09.010 33002645

[B5] CotelliM.CalabriaM.ManentiR.RosiniS.ZanettiO.CappaS. F. (2011). Improved language performance in Alzheimer disease following brain stimulation. *J. Neurol. Neurosurg. Psychiatry* 82 794–797. 10.1136/jnnp.2009.197848 20574108

[B6] De RisioL.BorgiM.PettorrusoM.MiuliA.OttomanaA. M.SocialiA. (2020). Recovering from depression with repetitive transcranial magnetic stimulation (rTMS): A systematic review and meta-analysis of preclinical studies. *Transl. Psychiatry* 10:393. 10.1038/s41398-020-01055-2 33173042PMC7655822

[B7] Di LorenzoF.MottaC.BonnìS.MercuriN. B.CaltagironeC.MartoranaA. (2019). LTP-like cortical plasticity is associated with verbal memory impairment in Alzheimer’s disease patients. *Brain Stimul.* 12 148–151. 10.1016/j.brs.2018.10.009 30352737

[B8] Di LorenzoF.MottaC.CasulaE. P.BonnìS.AssognaM.CaltagironeC. (2020). LTP-like cortical plasticity predicts conversion to dementia in patients with memory impairment. *Brain Stimul.* 13 1175–1182. 10.1016/j.brs.2020.05.013 32485235

[B9] DongX.YanL.HuangL.GuanX.DongC.TaoH. (2018). Repetitive transcranial magnetic stimulation for the treatment of Alzheimer’s disease: A systematic review and meta-analysis of randomized controlled trials. *PLoS One* 13:e0205704. 10.1371/journal.pone.0205704 30312319PMC6185837

[B10] Drumond MarraH. L.MyczkowskiM. L.Maia MemóriaC.ArnautD.Leite RibeiroP.Sardinha MansurC. G. (2015). Marcolin, transcranial magnetic stimulation to address mild cognitive impairment in the elderly: A randomized controlled study. *Behav. Neurol.* 2015:287843. 10.1155/2015/287843 26160997PMC4487699

[B11] FurtadoC. P.HoyK. E.MallerJ. J.SavageG.DaskalakisZ. J.FitzgeraldP. B. (2013). An investigation of medial temporal lobe changes and cognition following antidepressant response: A prospective rTMS study. *Brain Stimul.* 6 346–354. 10.1016/j.brs.2012.06.006 22784443

[B12] GangitanoM.Valero-CabréA.TormosJ. M.MottaghyF. M.RomeroJ. R.Pascual-LeoneA. (2002). Modulation of input-output curves by low and high frequency repetitive transcranial magnetic stimulation of the motor cortex. *Clin. Neurophysiol.* 113 1249–1257. 10.1016/s1388-2457(02)00109-812140004

[B13] HayasakaS.NakamuraM.NodaY.IzunoT.SaekiT.IwanariH. (2017). Lateralized hippocampal volume increase following high-frequency left prefrontal repetitive transcranial magnetic stimulation in patients with major depression. *Psychiatry Clin. Neurosci.* 71 747–758. 10.1111/pcn.12547 28631869

The article "The therapeutic efficacy of transcranial magnetic stimulation in managing Alzheimer’s disease: A systemic review and meta-analysis" was published in 2022. Journal: Front Aging Neurosci.

[B14] Health Quality Ontario (2016). Repetitive transcranial magnetic stimulation for treatment-resistant depression: A systematic review and meta-analysis of randomized controlled trials. *Ont. Health Technol. Assess.* 16 1–66.PMC480871927099642

[B15] JiaY.XuL.YangK.ZhangY.LvX.ZhuZ. (2021). Precision repetitive transcranial magnetic stimulation over the left parietal cortex improves memory in Alzheimer’s Disease: A randomized, double-blind, sham-controlled study. *Front. Aging Neurosci.* 13:693611. 10.3389/fnagi.2021.693611 34267648PMC8276073

[B16] JiangW.WuZ.WenL.SunL.ZhouM.JiangX. (2022). The efficacy of high- or low-frequency transcranial magnetic stimulation in Alzheimer’s Disease patients with behavioral and psychological symptoms of dementia. *Adv. Ther.* 39 286–295. 10.1007/s12325-021-01964-8 34716559

[B17] KiyoshigeE.KabayamaM.GondoY.MasuiY.InagakiH.OgawaM. (2019). Age group differences in association between IADL decline and depressive symptoms in community-dwelling elderly. *BMC Geriatr.* 19:309. 10.1186/s12877-019-1333-6 31722665PMC6854629

[B18] KochG.BonniS.PellicciariM. C.CasulaE. P.ManciniM.EspositoR. (2018). Transcranial magnetic stimulation of the precuneus enhances memory and neural activity in prodromal Alzheimer’s disease. *Neuroimage* 169 302–311. 10.1016/j.neuroimage.2017.12.048 29277405

[B19] KoyanoW.ShibataH.NakazatoK.HagaH.SuyamaY. (1991). Measurement of competence: Reliability and validity of the TMIG Index of Competence. *Arch Gerontol. Geriatr.* 13 103–116. 10.1016/0167-4943(91)90053-s15374421

[B20] LaneC. A.HardyJ.SchottJ. M. (2018). Alzheimer’s disease. *Eur. J. Neurol.* 25 59–70. 10.1111/ene.13439 28872215

[B21] LefaucheurJ. P.AlemanA.BaekenC.BenningerD. H.BrunelinJ.Di LazzaroV. (2020). Evidence-based guidelines on the therapeutic use of repetitive transcranial magnetic stimulation (rTMS): An update (2014-2018). *Clin. Neurophysiol.* 131 474–528. 10.1016/j.clinph.2019.11.002 31901449

[B22] LeocaniL.Dalla CostaG.CoppiE.SantangeloR.PisaM.FerrariL. (2020). Repetitive transcranial magnetic stimulation with H-Coil in Alzheimer’s Disease: A double-blind, placebo-controlled pilot study. *Front. Neurol.* 11:614351. 10.3389/fneur.2020.614351 33679572PMC7930223

[B23] LiX.QiG.YuC.LianG.ZhengH.WuS. (2021). Cortical plasticity is correlated with cognitive improvement in Alzheimer’s disease patients after rTMS treatment. *Brain Stimul.* 14 503–510. 10.1016/j.brs.2021.01.012 33581283

[B24] LiaoX.LiG.WangA.LiuT.FengS.GuoZ. (2015). repetitive transcranial magnetic stimulation as an alternative therapy for cognitive impairment in Alzheimer’s Disease: A meta-analysis. *J. Alzheimers Dis.* 48 463–472. 10.3233/jad-150346 26402010

The article "The therapeutic efficacy of transcranial magnetic stimulation in managing Alzheimer’s disease: A systemic review and meta-analysis" was published in 2022. Journal: Front Aging Neurosci.

[B25] LinY.JiangW. J.ShanP. Y.LuM.WangT.LiR. H. (2019). The role of repetitive transcranial magnetic stimulation (rTMS) in the treatment of cognitive impairment in patients with Alzheimer’s disease: A systematic review and meta-analysis. *J. Neurol. Sci.* 398 184–191. 10.1016/j.jns.2019.01.038 30735817

[B26] McInnesM. D. F.MoherD.ThombsB. D.McGrathT. A.BossuytP. M.CliffordT. (2018). Preferred reporting items for a systematic review and meta-analysis of diagnostic test accuracy studies: The PRISMA-DTA Statement. *Jama* 319 388–396. 10.1001/jama.2017.19163 29362800

[B27] MuellerJ. K.GrigsbyE. M.PrevostoV.PetragliaF. W.IIIRaoH.DengZ. D. (2014). Grill, Simultaneous transcranial magnetic stimulation and single-neuron recording in alert non-human primates. *Nat. Neurosci.* 17 1130–1136. 10.1038/nn.3751 24974797PMC4115015

[B28] NardoneR.TezzonF.HöllerY.GolaszewskiS.TrinkaE.BrigoF. (2014). Transcranial magnetic stimulation (TMS)/repetitive TMS in mild cognitive impairment and Alzheimer’s disease. *Acta Neurol. Scand.* 129 351–366. 10.1111/ane.12223 24506061

[B29] NguyenJ. P.SuarezA.KemounG.MeignierM.Le SaoutE.DamierP. (2017). Repetitive transcranial magnetic stimulation combined with cognitive training for the treatment of Alzheimer’s disease. *Neurophysiol. Clin.* 47 47–53. 10.1016/j.neucli.2017.01.001 28161090

[B30] PadalaP. R.BoozerE. M.LensingS. Y.ParkesC. M.HunterC. R.DennisR. A. (2020). Neuromodulation for apathy in Alzheimer’s Disease: A double-blind, randomized, sham-controlled pilot study. *J. Alzheimers Dis.* 77 1483–1493. 10.3233/jad-200640 32925060PMC7683089

[B31] PennisiG.FerriR.LanzaG.CantoneM.PennisiM.PuglisiV. (2011). Transcranial magnetic stimulation in Alzheimer’s disease: A neurophysiological marker of cortical hyperexcitability. *J. Neural. Transm (Vienna)* 118 587–598. 10.1007/s00702-010-0554-9 21207079

[B32] RabeyJ. M.DobronevskyE.AichenbaumS.GonenO.MartonR. G.KhaigrekhtM. (2013). Repetitive transcranial magnetic stimulation combined with cognitive training is a safe and effective modality for the treatment of Alzheimer’s disease: A randomized, double-blind study. *J. Neural. Transm (Vienna)* 120 813–819. 10.1007/s00702-012-0902-z 23076723

[B33] RainaP.SantaguidaP.IsmailaA.PattersonC.CowanD.LevineM. (2008). Effectiveness of cholinesterase inhibitors and memantine for treating dementia: Evidence review for a clinical practice guideline. *Ann. Intern. Med.* 148 379–397. 10.7326/0003-4819-148-5-200803040-00009 18316756

[B34] SterneJ. A. C.SavovićJ.PageM. J.ElbersR. G.BlencoweN. S.BoutronI. (2019). RoB 2: A revised tool for assessing risk of bias in randomised trials. *BMJ* 366:l4898. 10.1136/bmj.l4898 31462531

The article "The therapeutic efficacy of transcranial magnetic stimulation in managing Alzheimer’s disease: A systemic review and meta-analysis" was published in 2022. Journal: Front Aging Neurosci.

[B35] TalerV.PhillipsN. A. (2008). Language performance in Alzheimer’s disease and mild cognitive impairment: A comparative review. *J. Clin. Exp. Neuropsychol.* 30 501–556. 10.1080/13803390701550128 18569251

[B36] TeselinkJ.BawaK. K.KooG. K.SankheK.LiuC. S.RapoportM. (2021). Efficacy of non-invasive brain stimulation on global cognition and neuropsychiatric symptoms in Alzheimer’s disease and mild cognitive impairment: A meta-analysis and systematic review. *Ageing Res. Rev.* 72:101499. 10.1016/j.arr.2021.101499 34700007

[B37] TrungJ.HanganuA.JobertS.DegrootC.Mejia-ConstainB.KibreabM. (2019). Transcranial magnetic stimulation improves cognition over time in Parkinson’s disease. *Parkinsonism Relat. Disord* 66 3–8. 10.1016/j.parkreldis.2019.07.006 31300260

[B38] TurrizianiP.SmirniD.ManganoG. R.ZappalaG.GiustinianiA.CipolottiL. (2019). Low-frequency repetitive transcranial magnetic stimulation of the right dorsolateral prefrontal cortex enhances recognition memory in Alzheimer’s Disease. *J. Alzheimers Dis.* 72 613–622. 10.3233/jad-190888 31609693

[B39] VecchioF.QuarantaD.MiragliaF.PappaletteraC.Di IorioR.L’AbbateF. (2022). Neuronavigated magnetic stimulation combined with cognitive training for Alzheimer’s patients: An EEG graph study. *GeroScience* 44 159–172. 10.1007/s11357-021-00508-w 34970718PMC8811083

[B40] WangX.MaoZ.LingZ.YuX. (2020). Repetitive transcranial magnetic stimulation for cognitive impairment in Alzheimer’s disease: A meta-analysis of randomized controlled trials. *J. Neurol.* 267 791–801. 10.1007/s00415-019-09644-y 31760522

[B41] WuY.XuW.LiuX.XuQ.TangL.WuS. (2015). Adjunctive treatment with high frequency repetitive transcranial magnetic stimulation for the behavioral and psychological symptoms of patients with Alzheimer’s disease: A randomized, double-blind, sham-controlled study. *Shanghai Arch. Psychiatry* 27 280–288. 10.11919/j.issn.1002-0829.215107 26977125PMC4764002

[B42] ZhangF.QinY.XieL.ZhengC.HuangX.ZhangM. (2019). High-frequency repetitive transcranial magnetic stimulation combined with cognitive training improves cognitive function and cortical metabolic ratios in Alzheimer’s disease. *Journal. Neural Transm (Vienna)* 126 1081–1094. 10.1007/s00702-019-02022-y 31292734

[B43] ZhaoJ.LiZ.CongY.ZhangJ.TanM.ZhangH. (2017). Repetitive transcranial magnetic stimulation improves cognitive function of Alzheimer’s disease patients. *Oncotarget* 8 33864–33871. 10.18632/oncotarget.13060 27823981PMC5464918

